# The significance of exosomal RNAs in the development, diagnosis, and treatment of pancreatic cancer

**DOI:** 10.1186/s12935-021-02059-8

**Published:** 2021-07-09

**Authors:** Zheng Zhao, Guiping Zhao, Shuyue Yang, Shengtao Zhu, Shutian Zhang, Peng Li

**Affiliations:** Department of Gastroenterology, Beijing Friendship Hospital, Capital Medical University, No. 95 Yong’an Road, Xicheng District, Beijing, 100050 China

**Keywords:** Exosome, Exosomal RNAs, Pancreatic cancer, Biomarker

## Abstract

Exosomes are single-membrane, secreted organelles with a diameter of 30–200 nm, containing diverse bioactive constituents, including DNAs, RNAs, proteins, and lipids, with prominent molecular heterogeneity. Extensive studies indicate that exosomal RNAs (e.g., microRNAs, long non-coding RNAs, and circular RNAs) can interact with many types of cancers, associated with several hallmark features like tumor growth, metastasis, and resistance to therapy. Pancreatic cancer (PaCa) is among the most lethal cancers worldwide, emerging as the seventh foremost cause of cancer-related death in both sexes. Hence, revealing the specific pathogenesis and improving the clinical diagnosis and treatment process are urgently required. As the study of exosomes has become an active area of research, the functional connections between exosomes and PaCa have been deeply investigated. Among these, exosomal RNAs seem to play a significant role in the development, diagnosis, and treatment of PaCa. Exosomal RNAs delivery ultimately modulates the various features of PaCa, and many scholars have interpreted how exosomal RNAs contribute to the proliferation, angiogenesis, migration, invasion, metastasis, immune escape, and drug resistance in PaCa. Besides, recent studies emphasize that exosomal RNAs may serve as diagnostic and prognostic biomarkers or therapeutic targets for PaCa. In this review, we will introduce these recent insights focusing on the discoveries of the relationship between exosomal RNAs and PaCa, and the potentially diagnostic and therapeutic applications of exosomes in PaCa.

## Background

Pancreatic cancer (PaCa) is among the most common and devastating malignancies worldwide. Globally, there were reported cases 495,773 and reported deaths 466,003 from PaCa in 2020, with approximately as many deaths as cases due to its poor prognosis; it ranks, the seventh foremost cause of cancer-related death for both sexes [1]. PaCa is one of the highest case-fatality cancer types among all solid tumors, as the 5-year survival rate is only 10% [2, 3]. The poor prognosis of PaCa may be attributed to several factors, including a lack of typical symptoms, difficulties in early diagnosis, high metastatic potential, and resistance to conventional treatment. PaCa, which has no significant symptoms in the early stage, is commonly caught late, which causes a delay in treatment [4, 5]. In particular, existing methods, including surgical techniques, chemotherapy, radiation, and immunotherapy, each faces its own challenges, such as recurrence after resection, resistance to chemotherapy and radiation, and uncertainty whether the immunotherapy can be effective for the individual [6, 7]. Hence, it is urgently needed to identify the specific pathogenesis mechanism and facilitate early diagnosis.

## Introduction to exosomes

Exosomes, first recognized in the 1980s by Trams et al., are single-membrane, secreted organelles with a diameter of 30–200 nm [8, 9]. Exosomes are membrane-bound extracellular vesicles (EVs) that are produced in the endosomal compartment of most eukaryotic cells. Exosomes contain diverse bioactive constituents, including mRNAs, non-coding RNAs (ncRNAs), proteins, and lipids, with prominent molecular heterogeneity [10–13]. Exosomes are originate from double invagination of the membranes of plasma and endosome, and this process is a dedicated mechanism that refers to protein selection, RNA packaging, and EV release [14]. Endosomes form at the plasma membrane or the Golgi, which are membrane-delimited intracellular transport carriers. Once released, exosomes can extend a new paradigm of cell-to-cell communication by transferring those cargoes from donor cells to recipient cells [15]. It is widely documented exosomes are associated with both normal physiology and acquired pathological activities, including but not limited to reproduction, immunity, infection, and tumors [16–19]. As for tumor development, exosomes have diverse activities, such as formation of the tumor microenvironment (TME), initiation, proliferation, angiogenesis, and metastasis [20–22]. Furthermore, the molecular heterogeneity of exosomes has been observed among cancer patients and healthy individuals, and the cargoes and the amounts of exosomes created by the same cell may be dramatically different if educated with different treatments [23–25]. In theory, the heterogeneity of tumor cell-derived exosomes (TDEs) allows them to fulfill diagnostic functions. Cargoes of TDEs, such as microRNAs (miRNAs), long RNAs (lncRNAs), and circular RNAs (circRNAs), have been detected in PaCa and become novel non-invasive biomarkers for PaCa [26, 27]. Moreover, exosomes are emerging as therapeutic tools in several diseases, including PaCa [28, 29]. Therefore, we will summarize the biological activities of exosomal RNAs in the initiation and development of PaCa, and introduce the potential clinical applications of exosomes in PaCa.

## Formation, secretion, and uptake of exosomes (Fig. 1)

**Fig. 1:** Formation, secretion, and uptake of exosomes

Exosomes are nanosized EVs enriched in specific nucleic acids, lipids, proteins, and glycoconjugates [30]. Overall, exosomes originate from the first invagination of the plasma membrane, giving rise to early endosomes, and the sequential engulfment of cytoplasmic contents to form multivesicular bodies (MVBs). MVBs are named for their appearance, with a specialized subset of endosomes that contain many small vesicles inside the larger body. After fusion with plasma membrane, MVBs are released as intraluminal vesicles (ILVs) [31, 32]. First, the invagination of the cell membrane forms the early endosome, and in this process, the extracellular fluids and constituents (e.g., proteins, lipids, and other metabolites) can be internalized into the early endosome and the cell membrane proteins. Next, MVBs are derived from the subsequent inward invagination of the endosomal membrane, allowing cytoplasmic components to be engulfed into the endosomes and enrich the cargoes of ILVs. Endosomes are membrane-delimited intracellular transport carriers. Three main endosome compartments exist: early, late, and recycling endosomes. Early endosomes mature into late endosomes that subsequently fuse with lysosomes. Recycling endosomes are a sub-compartment of early endosomes that return material to the plasma membrane. Endosomes form at the plasma membrane or the Golgi. MVBs may fuse with lysosomes, and their cargoes will be degraded and recycled. Some MVBs fuse with the cell membrane and are transported into the extracellular milieu as exosomes [33, 34]. Such endosomes are called MVBs because of their appearance, with many small vesicles ILVs, inside the larger body. The ILVs become exosomes if the MVB merges with the cell membrane, releasing the internal vesicles into the extracellular space. Several proteins are indispensable in the formation of exosomes, including endosomal sorting complex required for transport (ESCRT), ALG-2 interacting protein X (ALIX), soluble *N*-ethylmaleimide-sensitive factor attachment protein receptors (SNAREs), tumor susceptibility 101 (TSG101), Rab GTPases, CD9, CD63, and CD81, some of which serve as markers of exosomes [15, 35, 36]. All these proteins play an integral role in the origin or biogenesis of EVs, and the precise functions of these proteins deserve further in-depth investigation. Once secreted into the extracellular milieu or bloodstream, exosomes can be recognized by recipient cells and then dock the cellular membrane, resulting in alterations in the behavior and phenotype of recipient cells [37]. The fate of the exosomes and their effects on recipient cells may vary because of their different cargoes, as the manners of uptake and utilization are complex. Upon docking at the plasma membrane, exosomes can fuse with the cellular membrane and deliver cargoes into the cytoplasm. In this process, recipient cells can internalize exosomes in several possible ways, including phagocytosis, macropinocytosis, caveolae-dependent endocytosis, and clathrin-dependent endocytosis [38, 39]. The different uptake pathways might rely on the types and physiologic state of recipient cells. For example, oncogenic KRAS expression can enhance exosome uptake efficacy by macropinocytosis in PaCa [40]. Cardiomyocytes can uptake circulating exosomal miRNAs via clathrin-mediated endocytosis, and human melanoma cells more readily rely on fusion with the plasma membrane for exosome uptake [41, 42]. After internalization, exosomes can deliver functional cargoes as the endpoint. In many cases, those exosomes can be released de novo by recipient cells, or the contents of exosomes are secreted into the endoplasmic reticulum and/or cytoplasm after the disintegration of intracellular vesicles such as endosomes or MVBs [43]. The different fates may depend on specific ligand receptors on the surface of exosomes and acceptor cells, but the exact mechanisms await further investigation.

## Current methods and challenges of the purification of exosomes

As critical mediators of intercellular crosstalk, exosomes exist in virtually all body fluids, and highly purified exosomes are indispensable for further structural and functional study [44]. However, the acquirement of high‐quality exosomes is still challenging due to exosome heterogeneity in the source, size, and content [45]. The *International Society for Extracellular Vesicles* has suggested that differential ultracentrifugation (DC) is the most frequently used method, with several other methods, such as density gradient ultracentrifugation (DGC), ultrafiltration (UF), precipitation, size-exclusion chromatography (SEC), and immunoaffinity capture [46]. We introduce the principles, advantages, and disadvantages of each of these conventional methods in Table 1. Although these conventional methods are widely available, several problems exist, such as labor- and time-consuming process, co-existence with impurities, and potential risk of exosomal damage. These disadvantages make it challenging to apply in clinical practice, especially for point-of-care testing (POCT). Recently, microfluidic techniques and aptamer-based magnetic techniques have been introduced as novel strategies of exosomal purification, which may provide compensation for the limitations of conventional methods [47, 48]. Microfluidic devices, including physical property-based methods, immune-chips capture, and comprehensive separation, have been developed for exosome purification [49, 50]. Compared with conventional methods, microfluidic techniques have apparent strengths, such as smaller sample volumes, faster assay times, lower reagent volumes, and higher portability. However, several problems are still to be overcome, such as a lack of standardized protocol, further improvement in purity, and additional reduction in cost. Aptamer-based magnetic techniques have been reported to achieve the rapid capture, adequate enrichment, and safe release of exosomes [51]. Therefore, this exosome purification method can potentially be applied to further investigations of exosomes and clinical translation of diagnosis and therapeutics. Nevertheless, there is neither sufficient evidence on the stability nor enough aptamer selection, which has limited the broad adaptability of their applications.

**Table 1:** The principles, advantages, and disadvantages of conventional methods of exosomal purification

Method	Principle	Advantage	Disadvantages
DC	By sequential increase in the centrifugal force, exosomes can be purified according to size and density	Suitable for large-volume samples Applied to purifying Exosomes from cell medium, plasma, and urine Relative technical simplicity	Time and labor cost Expensive equipment Damage due to centrifugal forces Large sample volumes requirement A mix of protein aggregates and lipoproteins
DGC	With the sample added to the medium of specific density, exosomes can be purified from multiple contaminants by density, mass, and size	Higher purity than that of DC	Same as those of DC
UF	By using a nanomembrane with a specific pore size and molecular weight cut-off, exosomes can be purified according to size or molecular weight	Saved time and labor consumption Fewer instruments cost Reduced technical difficulty	Damage to exosomes A mix of impurities with similar size or molecular weight Loss of small size exosomes Membrane blocking
SEC	By using a porous stationary phase with a specific pore size, exosomes can be purified while crossing the pores	Reservation of the biological activity and structural integrity of exosomes Saved time and labor consumption High yields Good reproducibility for purification from serum, plasma, ascites, and saliva	A mix of albumin and lipoproteins Special equipment
Precipitation	With precipitation reagents added to the sample and incubation, exosomes can be enriched from serum or plasma	Ease of use High yield Lower instruments requirements Commercialization of precipitation kits	A mix of lipoproteins, proteins, and ectosomes Difficult to remove the reagents from exosomes
Immunoaffinity capture	With antibodies that can recognize specific proteins deposited on the surfaces of magnetic beads, exosomes can be purified while modified beads capture the exosomal proteins	High purity Commercialization of immunoaffinity capture kits Able to separate sub-population exosomes	Damage due to elution Expensive reagents Low capacity A mix of apoptotic bodies and microvesicles

*DC* differential ultracentrifugation, *DGC* density gradient ultracentrifugation, *UF* ultrafiltration, *SEC* size-exclusion chromatography

## Exosomal RNAs play pivotal roles in PaCa development and progression (Fig. 2)

**Fig. 2:** Exosomal RNAs play pivotal roles in Paca development and progression

Exosomes are loaded with multiple cargoes, such as RNAs, DNAs, proteins, and lipids, and thus the delivery of exosomes plays pivotal roles in diverse physiological and pathophysiological processes [9]. Investigations into the correlation between exosomes and tumors have progressed rapidly, which has led to numerous significant discoveries in the development and progression of tumors, including proliferation, apoptosis, angiogenesis, migration, invasion, metastasis, immune escape, and drug resistance [20, 52–56]. Among these, exosomal RNAs have been intensively studied due to their essential roles in regulating all aspects of tumor metabolism and function [57]. In PaCa, cancer cells can be influenced by exosomal RNAs secreted from neighboring cancer cells or other cells, such as pancreatic stellate cells (PSCs), tumor-associated macrophages (TAMs), and cancer-associated fibroblasts (CAFs) [58–60]. Exosomal RNA delivery ultimately modulates the various features of PaCa, and many scholars have interpreted the role of exosomal RNAs in PaCa development and progression (Table 2).

**Table 2:** Exosomal RNAs involved in the development and progression in PaCa

RNA Type	Molecules	Origin	Effects	Targets	Refs.
miRNA	miRNA-222	TDEs	Proliferation ↑ Invasion ↑	p27/Akt	[61]
	miRNA-501-3p	TAMs	Tumorigenesis ↑ Metastasis ↑	TGFBR3/ TGF-β	[62]
	miRNA-5703	PSCs	Proliferation ↑	CMTM4/PI3K/Akt	[63]
	miRNA-3607-3p	NK cells	Proliferation ↓ Migration ↓ Invasion ↓	IL-26	[64]
	miRNA-1231	BM-MSCs	Proliferation ↓ Migration ↓ Invasion ↓	Not mentioned	[65]
	miRNA-126-3p	BM-MSCs	Proliferation ↓ Migration ↓ Invasion ↓	ADAM9	[66]
	miRNA-27a	TDEs	Angiogenesis ↑	BTG2	[68]
	miRNA-10a-5p	CAFs	Migration ↑ Invasion ↑	VDR	[71]
	miRNA-21	CAFs	Migration ↑ Invasion ↑	Not mentioned	[72]
	miRNA-221	CAFs	Migration ↑ Invasion ↑	NF-κ B/KRAS	[72]
	miRNA-21-5p	PSCs	Proliferation ↑ Migration ↑	Not mentioned	[73]
	miRNA-451a	PSCs	Proliferation ↑ Migration ↑	Not mentioned	[73]
	miRNA-125b-5p	TDEs	Migration ↑ Invasion ↑ EMT ↑	MEK2/ERK2	[85]
	miRNA-301a	TDEs	Migration ↑ Invasion ↑ EMT ↑	PTEN/PI3Kγ	[86]
	miRNA-203	TDEs	Immune Escape ↑	TNF-α/IL-12/TLR4	[94]
	miRNA-212-3p	TDEs	Immune Escape ↑	RFXAP/ MHC II	[95]
	miRNA-210	TDEs	GEM-resistance ↑	mTOR	[99]
	miRNA-106b	CAFs	GEM-resistance ↑	TP53INP1	[100]
	miRNA-365	TAMs	GEM-resistance ↑	NTP/CDA	[101]
	miRNA-155	TDEs	GEM-resistance ↑	SOD/CAT/DCK	[103]
	miRNA-194-5p	TDEs	Radiotherapy-resistance ↑	E2F3	[105]
lncRNA	UCA1	TDEs	Angiogenesis ↑	miRNA-96-5p/AMOTL2	[69]
	SBF2-AS1	TAMs	Migration ↑ Invasion ↑ Metastasis ↑	miRNA-122-5p/XIAP	[74]
	HULC	TAMs	EMT ↑ Invasion ↑ Migration ↑	Not mentioned	[75]
	NONHSAT105177	TDEs	Proliferation ↓ Migration ↓ EMT ↓	Clusterin	[76]
	Sox2ot	TDEs	Invasion ↑ Metastasis ↑ EMT ↑	miRNA-200 family/ Sox2	[77]
circRNA	PDE8A	TDEs	Invasion ↑	miRNA-338/MACC1/MET	[78]
	IARS	TDEs	Metastasis ↑	HUVECs	[79]
	hsa_circ_0002130	TDEs	Radiotherapy-resistance ↑	Not mentioned	[106]

## Proliferation and angiogenesis

Proliferation and angiogenesis are crucial elements in the rapid growth and development of PaCa, contributing to the severity of the disease. Recently, researchers have demonstrated that exosomal RNAs regulate the proliferation of PaCa by influencing the expression of multiple genes and activating different signaling pathways. For instance, tumor-derived exosomal miRNA-222 was reported to promote the proliferation and invasion of PaCa cells via increasing p27 phosphorylation by activating Akt signaling [61]. In another study, TAM-derived exosomal miRNA-501-3p was found to increase tumorigenesis and metastasis through the transforming growth factor-β receptor 3 (TGFBR3) -mediated TGF-β signaling pathway [62]. In addition, PSC-derived exosomal miRNA-5703 was found to promote PaCa proliferation by downregulating CKLF like MARVEL transmembrane domain-containing protein 4 (CMTM4) and activating the PI3K/Akt pathway [63]. Although the origins and targeted signaling pathways vary, exosomal RNAs appear to play multiple crucial roles in PaCa proliferation. In contrast, some exosomal RNAs have opposite effects, such as inducing apoptosis. In this regard, Sun et al. found that natural killer (NK) cell-derived exosomal miRNA-3607-3p inhibits PaCa proliferation, migration, and invasion by targeting IL-26 [64]. Additionally, exosomal miRNA-1231 and miRNA-126-3p, secreted by bone marrow mesenchymal stem cells (BM-MSCs), are implicated in inhibiting the proliferation, migration, and invasion of PaCa cells [65, 66]. Likewise, miRNA-126-3p promotes the apoptosis of PaCa cells by silencing of a disintegrin and a metalloproteinase 9 (ADAM9)[66]. In summary, exosomal RNAs are capable of both promoting and inhibiting carcinogenesis depending on their different mechanisms. As a unique link between proliferation and apoptosis, angiogenesis is deeply involved in tumor growth and metastatic dissemination [67]. Several exosomal RNAs have been identified to be associated with angiogenesis in PaCa. Tumor-derived exosomal miRNA-27a was found to promote angiogenesis in PaCa via B-cell translocation gene 2 (BTG2) [68]. Additionally, hypoxic tumor-derived exosomal lncRNA urothelial cancer-associated 1 (UCA1) was shown to promote angiogenesis via miRNA-96-5p/AMOTL2 (angiomotin-like 2) in PaCa [69]. Above all, these studies show how exosomal RNAs with different functions from diverse origins can affect tumor growth. However, we cannot attribute the poor prognosis only to the presence of highly proliferative cancer cells, as the prognosis is affected by multiple factors, including migration, invasion, metastasis, immune escape, and drug resistance.

## Migration, invasion, and metastasis

PaCa is characterized by aggressive features including migration, invasion, and metastasis, which always cause early treatment failure [58]. With these features, cancer cells are able to move to adjacent and distant areas and even settle in secondary tissues and organs [70]. As mentioned above, several exosomal RNAs (including miRNA-222, miRNA-501-3p, miRNA-5703, miRNA-3607-3p, miRNA-1231, miRNA-126-3p) have been found to promote or inhibit PaCa migration, invasion, and metastasis [61–66]. Additionally, CAF-secreted exosomal miRNA-10a-5p was found to promote migration and invasion in PaCa cells, while activating vitamin D receptor (VDR) signaling could inhibit these supportive effects on PaCa cells [71]. Similarly, CAF-derived exosomal miRNA-21, miRNA-221, PSC-derived exosomal miRNA-21-5p, and miRNA-451a were reported to confer aggressive features in PaCa cells [72, 73]. In the context of inhibitory effects, NK cell-derived exosomal miRNA-3607-3p was reported to inhibit the migration and invasion of PaCa cells by directly targeting IL-26 [64]. In addition, BM-MSCs-derived exosomal miRNA-1231 and miRNA-126-3p were also indicated to act inhibitory roles of the migration and invasion of PaCa cells [65, 66]. Interestingly, exosomal lncRNAs and circRNAs seem to be more active in migration, invasion, and metastasis than that in proliferation in PaCa. Tumor-derived exosomal lncRNA SBF2 antisense RNA 1 (SBF2-AS1), highly upregulated in liver cancer (HULC), NONHSAT105177, SOX2 overlapping transcript (Sox2ot), circRNA phosphodiesterase 8A (PDE8A), and isoleucyl-tRNA synthetase (IARS) have already been reported to affect the migration, invasion, and metastasis of PaCa cells [74–79]. Naturally, exosomal RNAs can also act as suppressive factors, as mentioned above. Thus, exosomal RNAs can act as major regulators of migration, invasion, and metastasis, promoting (or inhibiting) the progression of PaCa. Moreover, epithelial–mesenchymal transition (EMT) is a special biological process involved in the migration, invasion, and metastasis [80]. In this process, in which epithelial cells become mesenchymal cells via loss of cell polarity and gain of molecular alterations [81].EMT is characterized by the loss of epithelial E-cadherin and the acquisition of mesenchymal markers such as N-cadherin, fibronectin, and vimentin [82–84]. Recently, several exosomal RNAs have been reported to promote EMT in PaCa [29]. For instance, tumor-derived exosomal miRNA-125b-5p was found to be upregulated in highly invasive PaCa cells, facilitating migration, invasion, and EMT via the activation of MEK2/ERK2 signaling [85]. In addition, exosomal miRNA-301a, lncRNA HULC, and NONHSAT105177 were also reported to contribute to EMT in PaCa [75, 76, 86]. Above all, we believe that these findings will be of great value if these factors are applied as targets for therapeutic intervention.

## Immune escape

The immune system is a complicated network of diverse cells and biomolecules that prospect the body against infection, cancer, and other harmful circumstances. Gene mutations and the abnormal proliferation of cancer cells can produce different types of antigens; these antigens allow the detection and elimination of cancer cells by a large variety of immune response factors, preventing potential malignant transformation. Exosomes have been previously well studied in the context of the immune response, and scholars have proposed many mechanisms that explain how cancer cells promote immune escape and cancer development [18, 87, 88]. Several studies have pointed out that tumor-derived exosomes realized immune escape by inhibiting the activation of immune cells, causing a functional loss in immune responses[89–92]. Dendritic cells (DCs) serve as the most critical antigen-presenting cells (APCs) of the human immune system, and they function by promoting the expression of Toll-like receptors (TLRs) and generating multiple interleukins (ILs). Among TLRs, TLR4 exhibits a powerful antitumor effect [93]. In PaCa, tumor-derived exosomal miRNA-203 was reported to downregulate TLR4 and downstream tumor necrosis factor α (TNF-α) and IL-12 in DCs, which may help PaCa cells achieve immune escape [94]. In another study, tumor-derived exosomal miRNA-212-3p was found to inhibit the expression of RFX-associated protein (RFXAP), which decreased the expression of major histocompatibility complex class II (MHC II) and mediated the immune tolerance of DCs [95]. These findings infer that exosomal RNAs can harbor functional immune activity, allowing PaCa cells to escape immune surveillance. However, relative to that in other research areas, our knowledge about how exosomes help cancers cells escape the immune system in PaCa is still limited, and additional work is needed to address this issue. Deeper insight into the relationship between exosomes and immune escape is likely to be beneficial for the identification of potential biomarkers and the development of therapeutics.

## Drug resistance

Systemic chemotherapy combinations, including gemcitabine (GEM) plus other drugs, are still the cornerstone of treatment for advanced PaCa [3], while drug resistance remains a severe challenge in the context of antitumor therapy. To our knowledge, cancer cells can develop drug resistance via enhanced DNA repair, altered membrane transport, defective apoptotic pathways, etc. [96]. The effect of exosomes in the process cannot be ignored. In normal cells, exosomes are responsible for the transport of many cargoes from one cell to another. Studies have demonstrated that, once drug-resistant cancer cells develop, exosomes loaded with so-called “anti-chemotherapy” information can confer drug resistance to sensitive cells [97, 98]. In PaCa, several exosomal RNAs have been discovered to play essential roles in drug resistance. For example, exosomes derived from GEM-resistant PaCa cells were found to enhance the drug resistance of other cancer cells by delivering miRNA-210 [99]. Another study indicated that CAF-derived exosomal miRNA-106b promoted PaCa GEM-resistance via tumor protein 53-induced nuclear protein 1 (TP53INP1) [100]. Likewise, the delivery of miRNA-365 in TAM-derived exosomes was shown to potentiate the GEM-response in PaCa[101]. Notably, with a series of successive validation studies, tumor-derived exosomal miRNA-155 was proven to be a vital related to GEM-resistance [102, 103]. These studies highlight the relationship between exosomal RNAs and GEM-resistance that exosomal RNAs can accelerate the acquisition of GEM-resistance and mitigate the cell-killing effect. In addition to newer therapeutic strategies, chemotherapy and radiotherapy still have considerable prospects for PaCa [104]. Similar to their regulatory roles in drug resistance, exosomal RNAs can also impact the outcome of radiotherapy. It has been reported that dying post-radiotherapy PaCa cells can deliver exosomal miRNA-194-5p to potentiate cell repopulation survival by modulating the expression of E2F transcription factor 3 (E2F3) [105]. In another study, exosomal hsa_circ_0002130 was considered to modulate cancer cell repopulation after radiation [106]. Overall, exosomal RNAs are related to the emergence of both drug resistance and radiotherapy resistance, and we believe that novel treatments targeting exosome‐specific therapeutic resistance markers will be developed soon.

## Exosomal RNAs as potential biomarkers for PaCa

With very few specific symptoms in the early period, PaCa is often diagnosed in an advanced stage, which leads to a high fatality rate [107]. Traditional imaging examinations, such as ultrasound, CT, and MRI, are widely used in the clinical evaluation of PaCa. Although CA-199 is the only FDA-approved biomarker of PaCa, its accuracy is far from satisfactory due to the poor sensitivity at an early stage and the relatively low specificity overall [108–110]. Therefore, a more precise method is urgently needed for non-invasive diagnosis. As mentioned earlier, exosomes are enriched with biological cargoes, so they have gained interest as potential biomarkers for the early diagnosis of multiple malignancies [111]. Among these, exosomal RNAs are emerging as novel biomarkers for PaCa (Table 3). Accumulated evidence has revealed that exosomal RNAs can be more valuable in diagnosis than peripheral blood-free RNA as they have several advantages: exosomes can prevent RNAs from being degraded via RNases; exosomal RNAs are more closely associated with those of the original cells; and there is a higher concentration of RNAs in exosomes, which can yield more information [112–114].

**Table 3:** Exosomal RNAs as biomarkers for Paca

RNA Type	Molecules	Origin	Potential functions	Refs.
miRNA	miRNA‑21	Peripheral blood	Early diagnosis/tumor stage/survival evaluation	[116–119]
	miRNA-210	Peripheral blood	Early diagnosis/tumor stage	[116]
	miRNA-10b	Peripheral blood	Early diagnosis	[117, 120]
	miRNA-1246	Peripheral blood	Early diagnosis	[121]
	miRNA-451a	Peripheral blood	Tumor stage/survival evaluation	[122]
	miRNA-222	Peripheral blood	Tumor stage/survival evaluation	[61]
	miRNA-4525	Portal vein blood	Recurrence prediction/survival evaluation	[124]
	miRNA-451a	Portal vein blood	Recurrence prediction/survival evaluation	[124]
	miRNA-21	Portal vein blood	Recurrence prediction/survival evaluation	[124]
	miRNA-21	Pancreatic juice	Early diagnosis	[125]
	miRNA-155	Pancreatic juice	Early diagnosis	[125]
	miRNA-1246	Salivary	Early diagnosis	[126]
	miRNA-4644	Salivary	Early diagnosis	[126]
lncRNA	Sox2ot	Peripheral blood	Tumor stage/survival evaluation	[77]
	HULC	Peripheral blood	Early diagnosis	[75]
	CRNDE	Peripheral blood	Early diagnosis	[136]
	MALAT-1	Peripheral blood	Early diagnosis	[136]
circRNA	PDE8A	Peripheral blood	Tumor stage/survival evaluation	[78]
	IARS	Peripheral blood	Tumor stage/survival evaluation	[79]
mRNA	WASF2	Peripheral blood	Early diagnosis/tumor stage/	[139]
	GPC1	Peripheral blood	Early diagnosis/tumor stage/	[140]

Among all exosomal cargoes, exosomal miRNAs are currently regarded as the most promising biomarkers because of their abundance and easy accessibility, indicating that they can be used as potential diagnostic tools; in addition, they are closely related to the outcome and recurrence of PaCa [115]. For example, several studies indicated that elevated exosomal miRNA‑21 levels can not only discriminate PaCa patients from healthy individuals and patients with other pancreatic diseases (e.g., chronic pancreatitis and intraductal papillary mucinous neoplasm) but can also help make an early diagnosis and evaluate tumor stage [116–119]. Moreover, other exosomal miRNAs, including miRNA-210, miRNA-10b, miRNA-451a and miRNA-1246, can be applied for the accurate and early diagnosis of PaCa [116, 117, 120, 121]. Notably, some exosomal miRNAs may be correlated with tumor recurrence or may even be independent prognostic factors for PaCa. For instance, high-level expression of exosomal miRNA-451a was found to be associated with an increased risk of cancer recurrence and poorer prognosis in PaCa [122]. Similarly, another study illustrated that a higher exosomal miRNA-222 level was one of the independent risk factors for PaCa patients, which could reflect an enlarged tumor size and a high TNM stage [61]. Apart from peripheral blood, exosomes collected from other bodily fluids may also contribute to PaCa diagnosis and prognosis prediction [123]. First, portal vein blood assessment of exosomal miRNA-4525, miRNA-451a, and miRNA-21 was confirmed to outperform peripheral blood assessment evaluating both disease-free survival and overall survival in PaCa patients [124]. Next, pancreatic juice exosomal miRNA-21 and miRNA-155 levels were shown to discriminate PaCa patients from chronic pancreatitis patients with better performance than blood-free exosomal miRNA and CA-199 levels [125]. In addition, salivary miRNA-1246 and miRNA-4644 were found to be promising biomarkers for PaCa [126]. Naturally, some researchers preferred combinations of multiple exosomal miRNAs or of exosomal miRNAs and other biomarkers to achieve better diagnostic yield in PaCa evaluation [127–129]. For example, a 3D microfluidic chip was designed to assess multiple exosomal biomarkers including surface proteins (CD81, EphA2, and CA-199) and exosomal miRNAs (miRNA-451a, miRNA-21, and miRNA-10b), and the accuracy of diagnosis and stage monitoring reached up to approximately 100% [130]. In another study, a six-miRNA panel, including let-7b-5p, miRNA-192-5p, miRNA-19a-3p, miRNA-19b-3p, miRNA-223-3p, and miRNA-25-3p, was introduced to facilitate early and noninvasive diagnosis of PaCa early from both serum and exosomal specimens [131]. In addition to improving diagnostic yield, researchers have introduced many new techniques to better detect exosomal RNAs [132–134]. Typically, Pang et al. invented a biosensor for one-step detection of exosomal miRNAs, which could be of great value for applying point-of-care cancer diagnosis in terms of accuracy and convenience [135]. Overall, we believe that exosomal miRNAs can certainly be applied to improve the diagnosis and prognosis of PaCa.

Although existing studies on exosomal lncRNAs, circRNAs, and mRNAs are limited compared to those on exosomal miRNAs, these molecules can also facilitate PaCa diagnosis. Some scholars have suggested that many exosomal lncRNAs serve as tumor biomarkers for PaCa. For example, high expression of Sox2ot in plasma exosomes was shown to predict late TNM stage and poor survival in PaCa patients [77]. Additionally, exosomal lncRNA HULC, colorectal neoplasia differentially expressed (CRNDE), and metastasis-associated lung adenocarcinoma transcript 1 (MALAT-1) were proven to have potential value in discriminating PaCa from other pancreatic diseases [75, 136]. Exosomal circRNAs are another kind of endogenous non-coding RNAs, and information on their importance in tumors and other diseases is emerging [137, 138]. In PaCa, both exosomal circRNA PDE8A and IARS are correlated with progression and prognosis [78, 79]. Studies have proposed that exosomal circRNAs will soon serve as novel biomarkers for PaCa. Moreover, exosomal mRNAs have recently been discovered as potential diagnostic biomarkers. For example, exosomal mRNA Wiskott-Aldrich syndrome protein Verprolin-homologous protein 2 (WASF2) provided excellent accuracy for distinguishing PaCa patients from healthy individuals, and distinguishing PaCa patients between stage 0/I/IIA and stage IIB/III/IV [139]. Another exosomal mRNA, glypican-1 (GPC1), provided excellent diagnostic performance in differentiating PaCa patients from patients with other pancreatic diseases and from healthy individuals, approaching 100% sensitivity and specificity [140].

Above all, exosomal RNAs are implied to be potential diagnostic and prognostic biomarkers for PaCa, as summarized in Table 3. With the emphasis on their potential value as PaCa biomarkers, we still need more experiments to verify their significance in the diagnosis and prognosis evaluation of PaCa. Ultimately, there remains an endless challenge to identify additional sensitive and specific exosomal biomarkers with the growth of our knowledge in the field of exosomes. Even though substantial advancements have been achieved, there is a long path ahead before discovering a perfect PaCa biomarker.

## The therapeutic value of exosomes in the treatment of PaCa

PaCa is one of the deadliest malignant tumors, and thus scientists have devoted significant efforts to seek better-targeted therapies [141, 142]. With the function of drug-payload delivery, exosomes have been increasingly explored as therapeutic agents [14, 143] (Fig. 3). Among all the drug cargoes loaded into exosomes, nucleic acids, especially miRNAs, small interfering RNA (siRNA), and hairpin RNA (shRNA), are the most favorite constructs [144]. Generally, those cargoes can be loaded into exosomes either before or after purification. In most cases, those cargoes can be loaded via incubation, transfection-based methods, or ultraviolet irradiation before purification [145–147]; whereas after purification, they can be loaded into exosomes by either physical methods (such as electroporation, plain incubation, and sonication), or chemical procedures (such as transfection kit, and mix with organic solvent) [148–152]. In contrast to previous drug carriers (e.g., liposomes), injected exosomes can be taken up by other cells more effectively and confer bioactive cargoes with less immune interference [23, 153, 154]. In addition, the heterogeneity of surface molecules on exosomes is more suitable for receptor-targeted features, which realize exosome-targeted therapy [155]. Hence, the therapeutic utilization of exosomes as nanocarriers has excellent potential. Currently, researchers are committed to engineering exosomes for the encapsulation of therapeutic ingredients. For example, Zhou et al. loaded purified exosomes with paclitaxel and gemcitabine monophosphate, and these exosomes showed extraordinary penetrating abilities and yielded excellent targeted chemotherapy efficacy [156]. It is well known that the KRAS gene is closely associated with cell proliferation, survival, and differentiation, so multiple studies have been conducted on the KRAS gene. Kamerkar et al. engineered exosomes to deliver siRNA or shRNA targeting KRAS in PaCa cells, which successfully inhibited tumor growth in mouse models and improved overall survival [40]. Likewise, Mendt et al. engineered exosomes with siRNA to target KRAS G12D, which increased the survival of several mouse models with Paca [157]. Moreover, the MD Anderson Cancer Center is leading a phase I clinical trial of MSC-derived exosomes with KRAS G12D siRNA to treat patients with KRAS G12D mutation–associated PaCa (NCT03608631).

**Fig. 3:** The potential of exosomes to act as therapeutic vehicles

Regardless of the exciting progress and these pioneering developments, using engineered exosomes as vehicles in the clinical treatment of PaCa still presents several challenges. First, it is not easy to ensure the homogeneity of the treatment effect of different exosomes, as the alignments probably having varying degrees of the same therapeutic implication. Subsequently, the present isolation techniques of exosomes are relatively suboptimal for the requirement of immunotherapy. Overall, increasing studies and achievements in exosome extraction techniques will facilitate the application of exosomes in the clinical treatment of PaCa.

## Conclusions and perspective

Above all, exosomes are special vesicles that mediate diverse biological functions. In this review, we highlighted the vital role of exosomal RNAs in PaCa. These discoveries may spark more studies to elucidate the pathogenesis and mechanism of PaCa, offering a new direction and important guidance for the diagnosis and treatment of PaCa. Nevertheless, the question remains whether observed biological activities, including the phenotypic and molecular alterations, can still persist under physiological conditions, which merits further validation.

Characterized by high specificity and minimally invasive nature, exosomal RNAs exhibit outstanding value as potential biomarkers for PaCa. However, large-scale studies are warranted to validate the clinical application of exosomal RNAs. To gain a greater value of the management of PaCa, exosomal RNAs may need to be more intensively studied to develop new utilities monitoring the outcome of therapy. In addition to simple prediction of recurrence and prognosis, if we can adjudicate a certain recurrence, judge the existence of metastasis, observe the therapeutic efficacy, or even determine the length of survival by just testing a specific exosomal RNA (or a set of exosomal RNAs), it will be of great convenience for both the patients and doctors. In terms of therapeutic applications of exosomes (represented by engineered exosomes), several major challenges remain for investigators, such as the evaluation of adverse effects and the identification of tolerated doses. In addition, it is vital to discover more active pharmaceutical ingredients, and identify their specific mechanisms, ensuring the homogeneity of in the treatment effect. Finally, back to the basics, the acquirement of high‐quality exosomes is still challenging, and several obstacles are still formidable, including standardization, improvements in throughput and purity, cost reduction, and increased exosome recovery. These problems, when resolved, will bring the bottom-up promotion to the application of exosomes to every degree.

## Data Availability

No new data were created or analyzed in this study. Data sharing is not applicable to this article.

## Abbreviations

PaCa: Pancreatic cancer
ncRNAs: Non-coding RNAs
EVs: Extracellular vesicles
TME: Tumor microenvironment
TDEs: Tumor cell-derived exosomes
miRNAs: MicroRNAs
lncRNAs: Long non-coding RNAs
circRNAs: Circular RNAs
MVBs: Multivesicular bodies
ILVs: Intraluminal vesicles
ESCRT: Endosomal sorting complex required for transport
ALIX: ALG-2 interacting protein X
SNAREs: Soluble *N*-ethylmaleimide-sensitive factor attachment protein receptors
TSG101: Tumor susceptibility 101
DC: Differential ultracentrifugation DGC: density gradient ultracentrifugation
UF: Ultrafiltration
SEC: Size-exclusion chromatography
POCT: Point-of-care testing
PSCs: Pancreatic stellate cells
TAMs: Tumor-associated macrophages
CAFs: Cancer-associated fibroblasts
PPP2R2A: Protein phosphatase 2 regulatory subunit Balpha
Akt: Protein kinase B
TGFBR3: Transforming growth factor-β receptor 3
PI3K: Phosphoinositide 3-kinase
CMTM4: CKLF like MARVEL transmembrane domain-containing protein 4
NK cell: Natural killer cell
BM-MSCs: Bone marrow mesenchymal stem cells
ADAM9: A disintegrin and a metalloproteinase 9
BTG2: B-cell translocation gene 2
UCA1: Urothelial cancer-associated 1
AMOTL2: Angiomotin-like 2
VDR: Vitamin D receptor
SBF2-AS1: SBF2 antisense RNA 1
HULC: Highly upregulated in liver cancer
Sox2ot: SOX2 overlapping transcript
PDE8A: Phosphodiesterase 8A
IARS: Isoleucyl-tRNA synthetizes
EMT: Epithelial–mesenchymal transition
MEK2: Mitogen-activated protein kinase kinase 2
ERK2: Extracellular signal-regulated kinase 2 PTEN: Phosphatase and tensin homolog
MACC: Metastasis-associated in colon cancer
MET: MET proto-oncogene, receptor tyrosine kinase
HUVECs: Human umbilical vein endothelial cells
DCs: Dendritic cells
APCs: Antigen-presenting cells
TLRs: Toll-like receptors
ILs: Interleukins TNF: Tumor necrosis factor
RFXAP: RFX-associated protein
MHC II: Major histocompatibility complex class II
GEM: Gemcitabine
mTOR: Mammalian target of rapamycin
TP53INP1: Tumor protein 53-induced nuclear protein 1
NTP: Nucleoside triphosphate
CDA: Cytidine deaminase
SOD: Superoxide dismutase 2
CAT: Catalase
DCK: Deoxycytidine kinase
E2F3: E2F transcription factor 3
CA-199: Carbohydrate antigen 199 XIAP: X-linked inhibitor of apoptosis protein
EphA2: Ephrin type-A receptor 2
IPMN: Intraductal papillary mucinous neoplasm
CP: Chronic pancreatitis
CRNDE: Colorectal neoplasia differentially expressed
MALAT-1: Metastasis-associated lung adenocarcinoma transcript 1
WASF2: Wiskott-Aldrich Syndrome Protein Family Member 2
GPC1: Glypican-1
siRNA: Small interfering RNA
shRNA: Small hairpin RNA
